The article "Potential Benefits of Music Therapy on Stroke Rehabilitation" was retracted in 2023. Reasons: signs of a paper mill; suspected computer-generated content; unreliable results or conclusions; concerns about the data.

# Potential Benefits of Music Therapy on Stroke Rehabilitation

**DOI:** 10.1155/2022/9386095

**Published:** 2022-06-15

**Authors:** Chengyan Xu, Zixia He, Zhipeng Shen, Fei Huang

**Affiliations:** ^1^Department of Neurosurgery, The Children's Hospital Zhejiang University School of Medicine, National Clinical Research Center for Child Health, Hangzhou, China; ^2^Department of Outpatient, The Children's Hospital Zhejiang University School of Medicine, National Clinical Research Center for Child Health, Hangzhou, China; ^3^Department of Science and Education, Hangzhou Women's Hospital, Hangzhou Maternity and Child Health Care Hospital, Hangzhou, China

## Abstract

Stroke is associated with a high rate of disability and mortality, and survivors are usually accompanied with dysphagia, aphasia, motor dysfunction, cognitive impairment, depression, and other complications. In the past decades, many studies have been conducted to reveal the pathogenesis and pathological mechanisms of stroke. Furthermore, treatment methods have been developed that contribute to the elevated survival rate of stroke patients. Early rehabilitation poststroke is starting to be recognized as important and has been receiving increasing attention in order to further improve the quality of life of the patients. As an emerging method of poststroke rehabilitation, music therapy can help attenuate dysphagia and aphasia, improve cognition and motor function, alleviate negative moods, and accelerate neurological recovery in stroke patients. This review helps summarize the recent progress that has been made using music therapy in stroke rehabilitation and is aimed at providing clinical evidence for the treatment of stroke patients.

## 1. Introduction

Stroke is a severe cerebrovascular disease that is associated with high morbidity, mortality, and disability. It seriously affects the daily lives of the patients and imposes a heavy burden on families and society. There are approximately 16 million people that suffer from stroke per year worldwide, of whom 5.7 million die and about 5 million become disabled [1]. The incidence of stroke in China is approximately 1000/100,000 per year, and the mortality rate is approximately 150/100,000 per year [2, 3]. Globally, China is a country that has the highest lifetime risk of stroke, as well as the heaviest disease burden. Stroke can cause dysphagia, aphasia, motor dysfunction, cognitive impairment, mood disorders, and other complications [4–7]. The neurological damage that is caused by stroke often cannot be completely recovered. With early intervention and rehabilitation, impaired neurological function can be restored to a certain extent at different stages of stroke, which mainly depends on the plasticity and functional reorganization of the brain [8–10]. Therefore, in order to conduct reasonable rehabilitation treatment for stroke patients, it is important to have the maximum curative effect, reduce the treatment cost, and alleviate the family and social burden of diseases.

The article "Potential Benefits of Music Therapy on Stroke Rehabilitation" was retracted in 2023. Reasons: signs of a paper mill; suspected computer-generated content; unreliable results or conclusions; concerns about the data.

Music therapy is a systematic treatment method that utilizes music elements as an intervention to improve patients' neurological function and mood status [11, 12]. Many studies have applied music therapy during rehabilitation of stroke, which has led to the achievement of a good effect [13, 14]. Due to its safety, it is low cost, convenient, simple, and easy to implement. It has good efficacy and is easily accepted by patients. Music therapy has started to receive more attention and application in stroke rehabilitation. This review summarizes and provides direction for the role of music therapy in the rehabilitation of stroke patients.

## 2. Music Therapy and Beneficial Effect on Neurological Disease

Music therapy mainly strengthens patients' perception of sound through rhythm and melody of music and improves patients' language understanding ability through lyrics and singing, as well as speech frequency and rhythm [15, 16]. The anatomical basis of music therapy is mainly the different processing of music by the brain hemispheres, with the left brain responsible for understanding lyrics and distinguishing rhythms, while the right brain deals with melody [17, 18]. Music therapy is comprised of two different types, the active type and the passive type. Active music therapy refers to when patients directly participate in singing, playing instruments, or moving with music during therapy. Passive music therapy, also known as sensory music therapy, allows patients to listen to familiar music. Passively listening to music has no special requirements, but it can create an environment that allows people to feel comfortable and safe [19–21]. For music selection, music with a strong sense of rhythm is chosen during active music therapy, while music is selected mainly based on personal preference during passive music therapy. Music selection and treatment plan design tend to be diverse, according to the degree of disease, the patient's age, gender, and cultural background [22–24].

Music therapy often exerts a beneficial effect on many neurological diseases, including neuropsychiatric disorders, chronic neurodegenerative diseases, epilepsy, and acute brain injury [25–27]. Many random clinical trials have been carried out and have provided strong evidence for the effectiveness of music therapy during disease remission. A clinical trial including 60 patients found that integration of music therapy with family recollection can help regulate physiological parameters. Hence, it is recommended to use this cost-effective therapy as a supplementary treatment for patients with traumatic brain injury [28]. Another study in which traumatic brain injury patients receive three months of neurological music therapy intervention has shown that there are enhanced executive functions and fine-grained neuroanatomical changes in the prefrontal areas [29]. Rhythmic auditory stimulation, as an important style of music therapy, can help improve the effect of gait training by reshaping the sensorimotor rhythms and strengthens frontal-temporal connectivity. Thus, this activity is able to sustain gait improvement in Parkinson's disease patients [30]. Furthermore, music therapy exerts a positive effect on the cognitive function of the patients with Alzheimer's disease and regulates factors that are related to sleep, mood, and quality of life [31, 32]. One of the most well-studied areas of music therapy is its application in neuropsychiatric diseases. Music therapy can help alleviate various types of anxiety, including preoperative anxiety [33, 34] and serious or long illness-induced anxiety [35, 36]. However, opposite results have demonstrated that music does not reduce anxiety among women receiving radiation therapy for cancer [37], which may be due to differences in the music therapy interval and initiation time. However, additional studies are required to discover the best path to decrease anxiety through music therapy. Music has been shown to relieve depressive symptoms across a number of clinical studies [38, 39]. A randomized controlled trial with 18 major depressive disorder patients who listen to 10 Hz beat-imbedded music therapy in combination with classical therapy showed no significant differences of depression scale, quality of life, and medication adherence compared to the control group [40]. Lu et al. revealed that psychiatric symptoms and depression status of schizophrenia patients are improved after using group music therapy, indicating that music therapy may be economical and an easily implemented method that improves mood and mental state [41]. It is important to note that during music therapy, the choice of music and the degree of the patients' illness all have an effect on treatment.

The article "Potential Benefits of Music Therapy on Stroke Rehabilitation" was retracted in 2023. Reasons: signs of a paper mill; suspected computer-generated content; unreliable results or conclusions; concerns about the data.

## 3. The Role of Music Therapy in the Rehabilitation Poststroke

### 3.1. Music Therapy Improves Dysphagia Poststroke

Dysphagia, a common complication of stroke, is mainly characterized by dysphonia, dysarthria, abnormal spontaneous cough, salivation, and choking after swallowing and is particularly common among the elderly [42, 43]. About 28%-67% of stroke patients tend to develop dysphagia [44], among which the incidence of dysphagia after stroke is 41% during the acute stage and 16% in the chronic stage [45]. Dysphagia can cause serious complications, including aspiration pneumonia, electrolyte disorders, and malnutrition. Additionally, stroke patients with dysphagia tend to develop psychological problems (i.e., fear of eating, anxiety, and depression), which seriously affect the patients' quality of life. Early rehabilitation plays an important role during the recovery of patients with dysphagia. Previous studies have discovered that swallowing training, acupuncture, electrical stimulation, transcranial magnetic stimulation, and other means can help stroke patients improve dysphagia and swallowing dysfunction [46–48].

In recent years, a large number of clinical studies have suggested that music therapy can effectively improve patients' dysphagia poststroke. A clinical study enrolled six stroke patients with mixed dysarthria. All patients underwent individual music therapy sessions. The duration of each session was 30 minutes, and 12 sessions in total were conducted. The maximum phonation time, fundamental frequency, average intensity, and sequential motion rates were increased after music therapy, indicating that music therapy can improve speech motor coordination, including respiration, phonation, articulation, resonance, and prosody [49]. Another study investigated the effect of vocal exercises and singing on intelligibility and speech naturalness among patients with acquired dysarthria, following traumatic brain injury or stroke. Each patient implemented 24 individual music therapy sessions within eight weeks. The content of music training included therapeutic singing using familiar songs, oral motor respiratory exercises, rhythmic and melodic articulation exercises, rhythmic speech cuing, and vocal intonation therapy. Functional speech intelligibility and speech naturalness were significantly improved after completing treatment, which demonstrates that timely and continuous vocal exercises and singing may help accelerate the recovery of speech after stroke [50]. A music-enhanced swallowing protocol was developed in a preliminary study conducted by Kim, among which eight stroke patients participated. After six sessions of therapy, oral motor control, laryngeal elevation, breathing, and swallowing functions of the patients were enhanced by improving oral motor control, which suggests the effectiveness of music therapy in stroke rehabilitation [51]. The number of participants in most current studies is small, and the data are from a single center. Multicenter large-scale clinical trials are needed in the future to further substantiate the effect of music therapy on the improvement of dysphagia after stroke.

The article "Potential Benefits of Music Therapy on Stroke Rehabilitation" was retracted in 2023. Reasons: signs of a paper mill; suspected computer-generated content; unreliable results or conclusions; concerns about the data.

### 3.2. Music Therapy Promotes Recovery of Motor Function Poststroke

Motor dysfunction is one of the most common complications following stroke, which manifests as numbness and weakness of the limbs and even paralysis or spasms [13, 52]. Motor dysfunction can seriously affect the quality of life and social participation of stroke patients. Rehabilitation of motor function after stroke is a progressive and dynamic process and mainly includes exercise training, drug therapy, and psychological counseling. A variety of innovative neurorehabilitation strategies are emerging tools that will help improve motor function after stroke [53]. Music therapy, as a novel method, provides a new way for the motor function rehabilitation of stroke patients. By listening to music or singing songs, it can help promote neural plasticity, regulate neural networks and signal transduction, and achieve the purpose of improving patients' motor function [54, 55].

Exercise training is an important rehabilitation measure that is utilized for the treatment of stroke patients with motor dysfunction. During treatment, music with a strong sense of rhythm is generally helpful for rehabilitation of motor function [56]. The motor system is sensitive to auditory stimulation, and music rhythms can excite motor neurons in order to cause the muscles to move in a natural and ideal way, improving the rhythm of action and quality of action completion. It also enhances the effect of exercise therapy in order to promote the recovery of the patients' limb motor function. Playing musical instruments or pulling an arm trainer with rhythmic music can help increase the frequency and fluency of finger movements, as well as upper extremity function [57–59], which can cause excitability changes in the motor cortex. In addition, studies have validated that adding sound feedback during exercise training can increase auditory input of the patients, which can help improve excitation of the motor cortex, promote brain function remodeling, and achieve auditory motor function integration [60]. Moreover, functional magnetic resonance imaging (MRI) suggests that one of the effects of music-supported therapy is task-dependent coupling of auditory and motor cortical areas [61].

As limb motor dysfunction in stroke patients can lead to gait impairment, many scholars focus on the impact of music therapy on gait training in stroke patients [62]. Patients that receive music motor feedback training have experienced a significant improvement in stride length and gait speed compared to routine gait training without music. Even after removing the external pacer, the gait of the patients may be improved to some extent through memory of music and rhythm [62]. In addition, studies have highlighted that patients that receive rhythmic auditory stimulation have significantly improved step velocity, stride frequency, symmetry and length, and balance function and trunk control, regardless of the type of rhythmic stimuli [63–66]. Previous studies have also discovered that rhythmic auditory stimulation can improve the gait of patients with acute, subacute, or chronic stroke [67, 68]. However, choosing the most appropriate music type, which involves considering rhythm, strength, and frequency, for stroke patients at different stages, remains to be further studied. The potential mechanism underlying music therapy-induced benefits have been extensively studied, and the results demonstrate that music therapy can enhance the effect of gait training by improving psychology and cognition, regulating neurotransmitter delivery, and enhancing the plasticity of the nervous system, as well as other mechanisms [69, 70].

The article "Potential Benefits of Music Therapy on Stroke Rehabilitation" was retracted in 2023. Reasons: signs of a paper mill; suspected computer-generated content; unreliable results or conclusions; concerns about the data.

The complex repair mechanism that is involved in limb dysfunction has not been clearly defined. Therefore, it is necessary to fully assess the degree and type of limb dysfunction among different stroke patients and explore its possible pathological mechanisms and risk factors. The period, course of treatment, intensity, and frequency of music therapy, as well as the combined rehabilitation therapy plan, are significantly different in current studies. Furthermore, various music therapy plans, evaluation index, and measurement scales are utilized in studies that are conducted across different centers. Therefore, standardized multicenter trials need to be carried out in the future to improve the clinical efficacy of music therapy in motor recovery after stroke. Additionally, the treatment plan should be rationally optimized to meet the individual needs of each patient.

### 3.3. Music Therapy Attenuates Aphasia Poststroke

Poststroke aphasia refers to a focal brain injury caused by stroke, leading to the destruction of cortical and subcortical structural networks within the dominant hemisphere of language. Thereby, it causes impaired or permanent loss of the production and understanding of language symbols, as well as language dysfunction during listening, speaking, reading, or writing [71, 72]. Aphasia is one of the important manifestations of neurological impairment after stroke. Aphasia has a high incidence during stroke and seriously affects the communication ability of the patients, aggravates neurological dysfunction, and brings great mental and economic burden to patients, families, and society. Medication, speech and language therapy, behavioral therapy, noninvasive brain stimulation, and other therapeutic strategies have been developed in order to decrease the incidence and alleviate the degree of aphasia poststroke [73–76].

The article "Potential Benefits of Music Therapy on Stroke Rehabilitation" was retracted in 2023. Reasons: signs of a paper mill; suspected computer-generated content; unreliable results or conclusions; concerns about the data.

Neuroimaging studies have discovered that there is an overlap between the brain regions that are activated during speech and singing, which suggests that singing and speech share some common neural pathways [77–79]. Music therapy is introduced during treatment of aphasia after stroke through carefully designed music experience, which stimulates the damaged brain language function area, regulates neuroplasticity changes within the language network, and promotes the recovery of speech function [80, 81]. Melodic intonation therapy (MIT) is the most popular and effective music therapy that is applied to aphasia poststroke (Table 1). It makes use of the patients' unimpaired singing ability to sing words and phrases during daily life with musical melody in order to improve patients' oral expression ability. Zhang et al. discovered that music therapy-based MIT can have a positive impact on the language function of stroke patients that suffer from aphasia in the Chinese population [82], and similar effects are observed in the Greek [83], Spanish [84], Italians [85], and other populations, which indicates that MIT therapy has a good therapeutic effect in the population across different regions. A systematic review, including six clinical trials involving 115 patients, was aimed at evaluating the effectiveness of music therapy in the recovery of language function in poststroke aphasia. The data reveal that MIT can improve functional communication, repetition, and naming of patients but does not improve comprehension [80]. Another recently published systematic review retrieves MIT-related literature, including 39 randomized controlled trials that focus on MIT intervention among patients with aphasia in the stroke recovery period. The results demonstrate the beneficial effect of MIT on language rehabilitation. However, further MRI studies have been recommended that can help determine the clinical evidence and intervention targets of MIT and help provide clear neural circuit prompts and predict models used for MIT intervention [86]. Lim et al. demonstrate that neurologic music therapy and speech language therapy are both effective treatments for poststroke aphasic patients during the chronic stage, and the former is effective in the subacute stage of stroke [87]. Therefore, it is important to choose the appropriate music therapy strategy for stroke patients at different stages, which is worthy of further study. Moreover, due to the variety of music intervention modes for aphasia, future studies need to further standardize intervention methods and clarify the measurement indicators (i.e., spontaneous speech, fluency, repetition, and naming) in order to clarify the effect of music therapy and develop a more appropriate treatment plan.

The article "Potential Benefits of Music Therapy on Stroke Rehabilitation" was retracted in 2023. Reasons: signs of a paper mill; suspected computer-generated content; unreliable results or conclusions; concerns about the data.

### 3.4. Music Therapy Enhances Cognitive Recovery Poststroke

Poststroke cognitive impairment refers to a series of cognitive damages with different symptoms and severity after stroke. Due to the influence of multiple factors, including etiology, type, location, and complications of stroke, the clinical manifestations of cognitive dysfunction after stroke are multiple and are associated with memory disorders, learning ability disorders, attention disorders, sensory and perceptual disorders, personality changes, and behavioral abnormalities [4, 88–91]. The manifestations of poststroke cognitive impairment are not single but actually often overlap and interact with each other in complex ways. Cognitive rehabilitation is the systematic use of medical and rehabilitation therapy to improve the daily living activities and delay further aggravation of cognitive impairment, daily living ability, and limb function of stroke. On the basis of evaluation of the patients' brain injury and cognitive function, the therapeutic activity system is formulated with a goal of improving cognitive function. Hence, the behavior pattern acquired before is reconstructed or a new correct cognitive pattern is established in order to compensate for changes in the brain and body. Current clinical treatment for poststroke cognitive impairment includes drug therapy, computer-assisted cognitive rehabilitation, physical therapy, noninvasive brain stimulation, and traditional Chinese medicine [92–95].

Recently, studies have shown that music therapy, regardless of playing a musical instrument or listening to music or singing, can improve cognitive function of stroke patients [96, 97]. Early music intervention for patients with stroke is beneficial for long-term plasticity changes of sensory and perceptual processes and promotes the recovery of cognitive function. Rosemann et al. have proposed that deficits in memory or attention do not contribute to music perception impairment after stroke [98]. Vocal music can help improve memory recovery after stroke, as vocal music engages extensive and bilateral networks within the brain observed by functional magnetic resonance imaging, which may stimulate structural and functional plasticity changes in brain neural networks that are crucial for emotional processing and memory [99, 100]. One clinical trial with 15 subjects was in a face-to-face interview after a four-week multimodal rehabilitation program, including music therapy. The participants stated that they had a positive experience with cognitive and emotional improvements [101]. Similarly, a prospective randomized study that was conducted in Greece enrolled 65 stroke patients and discovered that music-based exercise programs have beneficial effects on the mood status of stroke patients and that the combination of exercise training and music treatment with familiar music had a better recovery effect [102]. Interestingly, different types of music exposure have different effects on poststroke cognitive impairment. Audiobook listening has been found to be associated with a positive distraction from thoughts and worries. Furthermore, mindful music listening is tightly associated with relaxation and concentration and strengthened attentional control. Music listening is also correlated with increased activity, memory reminiscence, and positive mood [103]. Therefore, the forms of music or sound input should be selected according to the main symptoms and severity of cognitive dysfunction in order to achieve the best therapeutic effect.

The article "Potential Benefits of Music Therapy on Stroke Rehabilitation" was retracted in 2023. Reasons: signs of a paper mill; suspected computer-generated content; unreliable results or conclusions; concerns about the data.

## 4. Conclusion

Overall, studies have demonstrated that music therapy in rehabilitation of stroke can help improve dysphagia, enhance the effect of limb motor exercise training, promote speech function recovery, and improve cognitive impairment. The mechanism of neurologic functional recovery after stroke is complex, and existing rehabilitation techniques are mainly focused on limb motor therapy and the recovery of brain function on the damaged side. As the integrity of the human brain function depends on close contact and interaction between the hemispheres, poststroke rehabilitation should not only enhance the recovery of the brain function on the injured side but also pay attention to the contralateral side in order to stimulate the hemispheres connectivity, resulting in an improvement in the integration of the entire brain function. Music therapy can improve neurological function by enhancing the neuroplasticity and neural networks of the brain. However, specific neurobiological mechanisms remain to be further explored.

Thus far, the effect of music therapy on rehabilitation following stroke has been gradually confirmed in clinic, and the therapy is simple, safe, and easy to accept. However, the patients' number of current clinical studies is small, and large-scale randomized controlled trials are needed. Moreover, the potential mechanisms of music therapy, implementation process, outcome evaluation, and treatment mode need to be further studied. In addition, as a kind of rehabilitation method, music therapy has a long treatment cycle and high requirements for patient compliance. And at present, the whole world is still short of professional music therapists, which need to cultivate more qualified therapists through international cooperation and exchange.

The article "Potential Benefits of Music Therapy on Stroke Rehabilitation" was retracted in 2023. Reasons: signs of a paper mill; suspected computer-generated content; unreliable results or conclusions; concerns about the data.

## Figures and Tables

**Table 1:** The application of melodic intonation therapy (MIT) in aphasia poststroke.

Participants	Intervention of MIT	Evaluation	Findings	References
The intervention group (*n* = 20; 16 males, 4 females) and the control group (*n* = 20; 15 males, 5 females)	Intervention group receives MIT treatment for 30 min/day, five times a week for 8 weeks	Boston diagnostic aphasia examination, Hamilton anxiety scale, and Hamilton depression scale	MIT has a better effect in fluency, spontaneous naming, object naming, reaction naming, and sentence completing, with a time accumulation effect	[82]

A 63-year-old man, 10 years poststroke, presented with a mild to moderate nonfluent aphasia	Receives MIT treatment 50 min twice weekly and attends a 4 hr socialization program once per week	Apraxia battery for adults, and Boston diagnostic aphasia evaluation	Integration of MIT by adding musical elements improves speech and expressive language skills, combined with a group socialization program	[104]

20 stroke patients with poststroke nonfluent aphasia	Receives MIT treatment for 12 sessions over six weeks	Communicative activity log questionnaire, Boston diagnostic aphasia examination	MIT may have a beneficial effect on the communication skills of stroke patients with nonfluent aphasia	[84]

17 patients with chronic (>1 year) poststroke aphasia. 10 in the MIT group and 7 in the control group	Receives 6 weeks intensive MIT (5 h/week)	Aachen aphasia test, Amsterdam-Nijmegen everyday language test, and Sabadel story retell task	MIT shows limited and temporary effect, suggesting that MIT exerts better effect for chronic aphasia in earlier stages poststroke	[105]

Six patients with severe nonfluent aphasia poststroke	Receives melodic-rhythmic therapy (a modified MIT) treatment 4 days a week for 16 weeks, with sessions of 30-40 min	Aachen aphasia test	MIT significantly improves the ability of spontaneous speech	[85]

Three participants with chronic poststroke Broca's aphasia	Receives MIT treatment in hourly sessions, 3 days per week for 6 weeks	Percent correct information units in connected speech, number of correct syllables in the trained and nontrained sentences, and visual analog mood scales	Combination of rhythm and pitch induces the strongest generalization effect to nontrained stimuli and connected speech. No significant effect in motor-speech agility or mood	[106]

Two patients with nonfluent aphasia poststroke	rTMS therapy (consisted of 3 treatment sessions) followed by 40 min of MIT	Western aphasia battery, fMRI	One patient has improvement in verbal fluency and repetition of phrases, while the other patient has no significant improvement. Neural activity changes are observed in the left Broca's area and right Broca's homolog	[107]

27 participants with subacute severe nonfluent aphasia poststroke	Receives MIT treatment in hourly sessions, 5 h per week for 6 weeks	Aachen aphasia test, semantic association task	MIT treatment has an improvement in verbal communication and language repetition	[108]

A patient with severe nonfluent aphasia poststroke	Receives intensive adapted MIT, attending five, 1.5-hour treatment sessions per week for 16 weeks	fMRI, DTI, and speech and language tasks	MIT induces functional and structural changes in a right hemisphere fronto-temporal network	[109]

30 acute stroke patients with nonfluent aphasia, 14 in the control group, and 16 in the treatment group	Receives a 10 to 15 min MIT session	Western aphasia battery	Significant immediate improvements in speech output after one session of MMIT training	[110]
Six patients with nonfluent aphasia at least 1 year postonset of first ischemic stroke	Treatment sessions are administered one per day for 3 consecutive days. The stimulation period of tDCS lasts for 20 min and combines with 20 min MIT	Boston diagnostic aphasia examination, verbal fluency tests	Transcranial direct current stimulation plus MIT contributes to significant improvements in fluency of speech, by enhancing activity in a right hemisphere sensorimotor network for articulation	[111]

Six patients with nonfluent aphasia at least 1 year postonset of first left hemisphere stroke	Receives an intense fashion with 75–80 daily therapy sessions	MRI and DTI; behavioral tests include number of correct information units/min produced during spontaneous speech, picture descriptions, and descriptions of common procedures	MTI increases the number of arcuate fasciculus fibers and arcuate fasciculus volume and improves the speech outcome	[112]

The article "Potential Benefits of Music Therapy on Stroke Rehabilitation" was retracted in 2023. Reasons: signs of a paper mill; suspected computer-generated content; unreliable results or conclusions; concerns about the data.

## Data Availability

No data were used to support this study.
